The article "Construction of COVID-19 Epidemic Prevention and Control and Public Health Emergency Response System Based on Discrete Stochastic Mathematical Model" was retracted in 2023. Reasons: suspected computer-generated content; unreliable results or conclusions; lack of ethics approval or compliance; missing or withdrawn patient consent.

# Construction of COVID-19 Epidemic Prevention and Control and Public Health Emergency Response System Based on Discrete Stochastic Mathematical Model

**DOI:** 10.1155/2022/5693293

**Published:** 2022-04-13

**Authors:** Ying Yang, Liming Dong, Hua Rong, HongyuYang, Bingxin Liu

**Affiliations:** ^1^Department of Nursing, General Hospital of Taiyuan Iron & Steel Co., Ltd, Taiyuan, 030008 Shanxi, China; ^2^Department of Gynaecology and Obstetrics, General Hospital of Taiyuan Iron & Steel Co., Ltd, Taiyuan, 030003 Shanxi, China; ^3^Department of Nursing, Taiyuan Fourth People's Hospital, Taiyuan, 030053 Shanxi Province, China; ^4^Department of Nursing, Shanxi Cancer Hospital, Taiyuan, Shanxi 030013, China

## Abstract

This research was aimed at exploring the construction and evaluation method of the comprehensive emergency response system for public health emergencies under the COVID-19 (coronavirus disease 2019) epidemic situation based on discrete stochastic mathematical model. The response of the Centers for Disease Control and Prevention (CDCP) of Taiyuan city in the COVID-19 epidemic situation was taken as an example. A new discrete stochastic COVID-19 epidemic spread mathematical model which integrated public health intervention and input cases was proposed. The model was parameterized by multisource data, and the impact of different flow patterns on the risk of secondary outbreak was analyzed. The advantages and disadvantages of its emergency system construction were analyzed. Additionally, the improvement measures and suggestions for the existing problems were proposed. Results suggested that there was only one specialized disease prevention and control institution in Taiyuan, and there were only 11 centers for disease prevention and control, accounting for 6.2% (11/177) of the total in Shanxi Province. Through the analysis, it was found that the current public health emergency response system in Taiyuan city had imperfect management coordination mechanism, incomplete plan type, serious shortage of public health personnel, poor information communication efficiency, insufficient early warning efficiency of the epidemic detection system, and weak logistics material security links. Therefore, it was proposed to establish a sound coordination system of emergency health management and vigorously promote the construction of emergency health management institutions. Thus, a public health emergency management system integrating management coordination system, plan system, emergency team building system, material reserve management, and other functions was formed. The application of discrete stochastic mathematical model suggests that intermittent population flow and effective isolation of infected people in transient population can effectively reduce the risk of secondary outbreak. The system analysis here also provides theoretical basis for improving the construction of public health emergency response system in Taiyuan.

## 1. Introduction

The epidemic situation of coronavirus disease 2019 (COVID-19) caused by novel coronavirus (SARS-CoV-2) infection has occurred in Wuhan, China, since December 2019. Then, it quickly spread to the whole country and formed a major epidemic, which caused huge losses to people's lives and property, leading to a huge blow to the social economy. It is the largest public health emergency in China since the SARS epidemic in 2003. The state's process of epidemic prevention and control is a major test of the construction of a major infectious disease treatment system and the status of emergency mechanisms. It also exposes the weak links in the early research judgment, prediction, control, diagnosis, and treatment of the epidemic situation in response to public health emergencies in China.

Public health emergencies refer to sudden outbreaks of major infectious diseases, mass unexplained diseases, and major food and occupational poisoning, as well as other events that affect public health that have caused or may cause serious damage to society and public health [1, 2]. It has the characteristics of suddenness, hazard, accident, publicity, and internationality, as well as comprehensiveness and systematicity of handling. Its harm and destruction to society, national life, and property safety are comprehensive and multifaceted. Also, it will not only cause harm to the lives and health of the people but also cause psychological panic among the people. In severe cases, it will also cause social chaos and economic paralysis, affecting national defense security [3–5]. Since the outbreak of SARS in 2003, the backwardness of China's health emergency system has been exposed. Therefore, many scholars worldwide have increased their research on the construction of public health emergency response systems to improve the government's ability to respond to major public health emergencies and risks. Infectious disease dynamics is a mathematical model that reflects the dynamic characteristics of infectious diseases established by scholars according to the laws of population growth, disease occurrence, transmission, and development in the population, as well as relevant social factors. The qualitative and the quantitative analysis and numerical simulation can analyze the development process of the disease, reveal the epidemic law, predict the change trend, and analyze the causes and key of the epidemic.

The newly revised *International Health Regulations* in 2005 have aroused the attention of countries around the world on the construction of early emergency systems [6–8]. Based on the epidemic caused by the Ebola virus infection in West Africa from 2014 to 2016, Brooks et al. explored and established a functional incident emergency management system to improve the management capacity of countries to respond to the epidemic [9]. Chen and Zhang constructed a metamodeling framework for public health emergency management through analysis of domain characteristics and modeling needs. Also, they took the Ebola epidemic as an example to show that the framework is used for the management and control of infectious diseases and other public health emergencies [10]. Sun et al. have summarized the development trend of China's emergency management system for public health emergencies since 2012 after the SARS epidemic raged in 2003 [11]. Xie et al. investigated a response decision model for unconventional public health emergency under the scenario-response paradigm and the discrete event system theory framework. Also, they performed simulation and optimization. The results showed that the scheme can meet the needs of emergency response to public health emergencies [12]. It can be seen that many investigations worldwide have been conducted on the construction and evaluation of public health emergency management systems. However, the spread of the COVID-19 epidemic has a greater impact. As of the end of May 2020, the cumulative number of confirmed cases in the world has reached 5.93 million, and the number of deaths exceeded 370,000. At present, the epidemic situation is still in the global outbreak trend, and it has not yet been stably controlled. It has evolved into a major global public health crisis. The current research is still insufficient to control and manage the COVID-19 epidemic.

Therefore, for the shortcomings exposed by the Centers for Disease Control and Prevention (CDCP) of Taiyuan city in response to the epidemic situation, the existing problems in the public health emergency management system were analyzed. Thereby, improvement measures were proposed to ensure that in the public health emergency, it can respond to various emergency situations in a timely and efficient manner, reducing the harm caused by various emergencies to a minimum.

## 2. Methods

### 2.1. Discrete Stochastic Model

Based on the disease transmission mechanism, individual epidemiological status, and prevention and control measures, the total population can be divided into seven categories: susceptible (*S*), latent (*E*), infected (*I*), hospitalized (*H*), recovered (*R*), isolated susceptible (*S*_*q*_), and isolated suspect (*B*). The process is shown in Figure 1. The category of isolated suspect in tracking isolation is added, which includes two parts: the latent person of tracking isolation and the individual with similar clinical symptoms. Considering the small number of imported cases in Taiyuan in the early stage, compared with the deterministic model, the difference system with stochastic input is more suitable to describe the situation and describe the stochasticness of population statistics.

Since Wuhan implemented the city closure strategy on January 23, 2020, prevention strategies in other provinces have been strengthened. To describe the continuously strengthened control strategy and the increasing diagnosis rate, the contact rate, isolation rate, diagnosis rate, and recovery rate are assumed to be functions of time *t*. It is assumed that the contact rate *c*(*t*) is a decreasing function of time *t*, which is shown as follows:

(1) $$\begin{array}{c} c\left(t\right)=\left\{\begin{array}{c} c_{0},\text{Before January }23,2020\;\\ \left(c_{0}-c_{b}\right)e^{-r_{1}t}+c_{b},\text{Others} \end{array}\right.. \end{array}$$

*c*_0_ refers to the contact rate of the initial period (i.e., before January 23, 2020), *c*_*b*_ represents the minimum value of the contact rate under the current control strategy, that is lim_*t*⟶∞_ = *c*(*t*) = *c*_*b*_, and *r*_1_ indicates the rate at which the number of contacts decreases exponentially.

The isolation rate *q*(*t*) is defined as an increasing function of time *t*, which can be expressed as follows:

(2) $$\begin{array}{c} q\left(t\right)=\left\{\begin{array}{c} q_{0},\text{Before January }23,2020\\ \left(q_{0}-q_{m}\right)e^{-r_{2}t}+q_{m},\text{Others} \end{array}\right.. \end{array}$$

*q*_0_ represents the initial isolation rate of the latent individual, *q*_*m*_ suggests the maximum isolation rate under the current control strategy, that is lim_*t*⟶∞_ = *q*(*t*), and *r*_2_ denotes the exponential growth rate of the isolation rate. In addition, the transfer rate *δ*_*I*_(*t*) is also defined as an increasing function of time *t*. Therefore, the detection period 1/*δ*_*I*_(*t*) is a decreasing function of time *t*, which can be expressed as follows:

(3) $$\begin{array}{c} \frac{1}{\delta_{I}\left(t\right)}=\left\{\begin{array}{c} \frac{1}{\delta_{I}0},\text{Before January }23,2020\\ \left(\frac{1}{\delta_{I}0}-\frac{1}{\delta_{I}f}\right)e^{-r_{3}t}+\frac{1}{\delta_{I}f},\text{Others} \end{array}\right.. \end{array}$$

*δ*_*I*_0 is the initial diagnosis rate, *δ*_*I*_*f* indicates the fastest diagnosis rate, that is lim_*t*⟶∞_ = *δ*_*I*_(*t*) = *δ*_*I*_*f*, and *r*_3_ means the exponential reduction rate of diagnosis time. *T*_*c*_ is set as the time point for the implementation of strict control measures on January 23, 2020. Until January 29, 2020, there are no recovered cases in Taiyuan. Therefore, the recovery rate is 0 before January 29, 2020. Since February 7, 2020, the number of patients recovered has increased rapidly. Therefore, based on the actual situation, the recovery rate is defined as a piecewise constant function.

### 2.2. Construction of Public Health Emergency Management System

Since the SARS epidemic in 2003, Taiyuan has strengthened its emphasis on the construction of the public health emergency management system as well as increased its development and research. Also, the improvement of the scientific emergency system has been promoted, and the relevant emergency laws and regulations have been actively implemented.  Figure 2 shows the structure of the public health emergency management system in Taiyuan.

In terms of the emergency management coordination system, to effectively respond to public health emergencies, it is necessary to establish a perfect emergency coordination management mechanism and implement a unified command and dispatch. It is the guarantee for the overall deployment of human and material resources. It is manifested within the disease control agency, that is, the establishment of a health emergency office or the designation of a special agency responsible for the daily management and work of health emergency. Its basic responsibility is to guide and coordinate the emergency treatment of public health emergencies of disease control agencies and formulate emergency plans for public health emergencies, as well as guide and undertake public health emergencies for prevention preparation, monitoring and early warning, disposal and rescue, and analysis and evaluation [13].

In terms of the formulation of emergency plans for public health incidents, China has formulated corresponding disposal plans and technical solutions based on various public health incidents and infectious viruses that have occurred worldwide. These include general plans and 6 types of special plans. There are “emergency plans for public health emergencies for poisoning events,” “emergency plans for accidents and disasters,” “emergency plans for terrorist incidents,” “emergency plans for natural disasters,” “emergency plans for mass unknown diseases,” and “emergency plans for major infectious diseases” [14].

In terms of the emergency team building system, the state and the government have been vigorously cultivating health technology personnel in recent years. According to the existing public health emergency management system, a three-level on-site treatment team for public health incidents and a three-level health emergency response personnel system for cities, districts (counties), and streets (villages) have been established. At the same time, training and learning of public health theoretical knowledge are regularly organized within the city [15].

In terms of the monitoring system, emergency monitoring capabilities play an important role in identifying the causes of emergency response. Public health event early warning, epidemic situation information report, and epidemic situation proliferation detection management need the monitoring system to conduct statistical analysis of information, thereby carrying out prevention and response in time. The current emergency system has a hierarchical response to public health events and a rapid response detection mechanism. From time to time, exercises will be conducted to test the efficiency of emergency supplies of relevant public health institutions and the efficiency of linkage between different departments.

In terms of informatization construction, digital technologies such as big data, artificial intelligence, and cloud computing are continuously developing in recent years [16–18]. Building an informatized public health emergency management system has become an important part of governments at all levels effectively performing public service functions. In this epidemic prevention and control work, Taiyuan has also begun to build an infectious disease prevention and control information network system. The three-level infectious disease epidemic reporting, prevention, and control network system in cities, districts (counties), and streets (villages) has initially taken shape. Subordinate institutions can report relevant infectious disease information through this prevention and control network system. At the same time, superior institutions can get relevant information in a timely manner and grasp the regional distribution of the relevant epidemic situation.

In terms of material reserve management and infrastructure construction, professional medical rescue agencies and rescue teams are an important foundation for urban disaster emergency medical work [19, 20]. However, the basis of disaster emergency medical work in cities across China is weak. Except for a few areas such as Shanghai, most provinces, cities, and counties (cities, districts) have not established corresponding professional emergency medical teams. Also, they lack the ability and experience to deal with major emergencies. In addition, there is also a lack of emergency rescue materials and equipment reserves. The mobile hospitals for disaster emergency medical rescue have not been established, and corresponding material reserves are lacking [21].

### 2.3. Application of Existing Public Health Emergency Management System

In the process of handling the public health incident of the COVID-19 epidemic, Taiyuan adopts the existing public health emergency management system. The shortcomings and advantages of the existing management system are analyzed according to the application. For the applied data sources, the case data of the COVID-19 epidemic situation comes from the infectious disease surveillance system and case epidemiological investigation data in the *China Information System for Disease Control and Prevention*. The population data during the same period and the staffing of the disease prevention and control agencies in various districts and counties, as well as the basic situation of human resources, are derived from the Taiyuan Statistical Yearbook. The basic situation of health emergency management, the construction of the emergency plan system, the formation of the health emergency team and the staffing situation, and the situation of health emergency equipment and material reserves are investigated through questionnaires.

### 2.4. Statistical Analysis of Data

The Excel software is used to collect, input, and organize all statistics and survey data. The SPSS 26.0 statistical software is used to process the data and perform corresponding statistical analysis.

## 3. Results and Discussion

### 3.1. Information Construction of COVID-19 Epidemic in Taiyuan

According to the daily report data of the epidemic situation in Taiyuan CDCP, the information of close contacts was collected. Since the first case of infection of COVID-19 was confirmed on January 22, 2020, until February 20, 2020, the number of newly confirmed cases decreased to 0 by May 1, 2020, and another case was found on May 2, 2020. By the end of May, a total of 21 cases of infection had been confirmed, 0 cases died, and 21 cases were cured. The incidence rate was about 0.45/10 million, with a mortality of 0%.  Figure 3 shows the onset time curve of confirmed cases of the COVID-19 epidemic in Taiyuan.

As can be seen from Figure 4, the onset date of the first case in Taiyuan is January 22. Generally, the number of confirmed cases reported has grown slowly. As of May 2, 2020, the number of confirmed cases reported per day was up to 3. The confirmed cases in the whole city were basically imported cases. For example, the confirmed cases on May 2 were confirmed to be imported confirmed cases in Hubei Province through investigation and tracking. After close tracking and control, there were no new cases of infection in Taiyuan after that. The peak period of infection was from February 1 to February 10, during which 14 cases were diagnosed.

The regional distribution of confirmed cases of the COVID-19 epidemic in Taiyuan is shown in Figure 3.

From the distribution area of the epidemic in Figure 3, the virus spread is mainly concentrated in the central area of Taiyuan. Wanbailin District, Yingze District, and Xinghualing District are all central areas of Taiyuan and belong to the old city of Taiyuan. The population is dense, the mobility is high, and the probability of virus infection is high. There are 18 confirmed cases in these three districts and counties, accounting for 85.71% of the total number of confirmed cases in the city. However, there is one case that is uncertain for the source, accounting for 4.76% of the total number of confirmed cases in the city.

It can be seen that in this epidemic prevention and control process, there are many information statistics that are not accurate enough. Also, the contact and coordination of various departments are not sufficient, resulting in inefficient information communication during epidemic prevention and control. It is limited by the top-level system, conflicts of interest between departments, and other factors. With the difference in operation modes of various districts (counties) brought about by the reform of the primary medical and health system, information communication efficiency is relatively low during the prevention and control of the COVID-19 epidemic in Taiyuan. This phenomenon is particularly prominent in the early stage of the outbreak, resulting in inefficient handling of public health events. Therefore, the information network system should be built and used at present. Internet, big data, cloud computing, and other network information technologies should be applied more extensively to truly exert the technical role of network information technology in early detection of major epidemics.

### 3.2. Management Situation of Disease Prevention and Control Institutions in Taiyuan

According to the 2019 health statistics report of the Taiyuan Municipal Health Commission, as of the end of 2019, among the medical and health institutions in Taiyuan, there are 58 public hospitals, accounting for 0.49% (58/11930) of the whole country, and 43 private hospitals, accounting for 0.19% (43/22424) of the whole country. In terms of the number of beds, the number of beds in public hospitals is 13296 and that in private hospitals is 5634 (Table 1). Regarding the characteristics of upward concentration of health resources, it is also necessary to focus on reducing the utilization rate of beds, improving the technical level, increasing the ratio of beds and nurses, and avoiding the situation that public hospitals exceed the standard of bed size. Meantime, the bed size of county hospitals, grass-root medical and health institutions, and social hospitals should be increased.  Figure 5 show the statistics on the nature of medical institutions in Taiyuan.

Table 1 indicates that there is only one specialized disease prevention and control institution in Taiyuan, and the number of CDCPs is only 11, accounting for 6.2% (11/177) of the total number of Shanxi Province. Figure 4 suggests that the overall number of tertiary medical institutions in Taiyuan is small, and the number of social medical institutions accounts for a large proportion in the total number of medical institutions. On the one hand, social medical institutions are conducive to establishing a competitive mechanism, improving the service efficiency and quality, improving the medical service system, and forming mutual promotion between public medical institutions and nonpublic medical institutions. On the other hand, most of the current policies and regulations on the supervision of social medical institutions are relatively lagging behind the status quo, and a good industry atmosphere has not yet been established.

Although the country has paid more attention to the training of public health emergency response personnel in recent years, overall, the number of health institutions has not increased significantly. Also, the audience is relatively narrow, generally only involving district (county) health and epidemic prevention institutions, and street (village) level is rarely involved. It can be seen that the number of professional institutions in the public health emergency system in Taiyuan is insufficient. Also, after investigation, it is found that none of the city's disease control agencies set up an independently prepared health emergency department. After the outbreak of the COVID-19 epidemic, the governments of various districts and counties, the municipal health bureau, the municipal public security bureau, and the municipal food and drug health supervision bureau established the COVID-19 epidemic prevention and control headquarters in Taiyuan to coordinate and manage the epidemic prevention and control work.

### 3.3. Human Resources

Analysis of the data collected shows that there are 699 staff for personnel allocation in 16 disease prevention and control institutions in Taiyuan. Among them, the municipal CDCP has 161 professional technicians, accounting for 23.03%. There are 538 professional technicians in disease control agencies of districts and counties, accounting for 76.97%. The composition of academic qualifications and positional titles of the Centers for Disease Control and Prevention are shown in Figures 6 and 7.

It can be seen from Figures 4 and 5 that there are 15 masters, accounting for 2.15%. The educational background is mainly junior college and technical secondary school, accounting for 26.90% and 32.62%, respectively. There are 99 people with a junior college education or above in municipal disease control institutions, accounting for 61.49%. The disease control institutions of district and county have 324 people under junior college education, accounting for 60.23%. There are 43 senior titles (6.15%), 183 intermediate titles (26.18%), 267 primary titles (38.20%), and 206 others (29.47%). It shows that the overall quality of the personnel of the disease prevention and control institutions in Taiyuan in this survey is not high. The educational background and positional title are low, especially the professional counterparts are few. In addition to the low penetration rate of higher education in China, the factor that cannot be ignored is that the staff engaged in disease prevention and control has a lower socioeconomic status than clinical medical staff. Northwest China is also a poor and backward region in the country, and it lacks attractiveness for outstanding talents. Therefore, it is necessary to vigorously strengthen the training of disease prevention and control as well as public health emergency personnel and improve the public health theory and practice of young and middle-aged teachers.

### 3.4. Emergency Plan Construction

Figures 8 and 9 show the infrastructure construction of CDCP in Taiyuan. Among the 11 CDCPs, the construction area per capita of Gujiao CDCP is the highest, up to 133.77 m^2^; the lowest is Jinyuan CDCP, which is 14.17 m^2^; among the county-level CDCPs, Qingxu CDCP has the lowest construction area, which is 37.71 m^2^.

However, the outbreak of the COVID-19 epidemic was sudden and significant. It is difficult to predict at that time that so many medical and health forces needed to be quickly invested in a short time. The relevant plan preparation is not enough to deal with the epidemic. Therefore, in the future, it is necessary to vigorously strengthen plan preparations for the handling of major public health emergencies. The establishment of emergency hospitals, personnel selection, and material preparation is not enough. The more important is the preparation of professional plans for public health emergency and medical rescue.

### 3.5. Monitoring System Construction

In the process of responding to the COVID-19 epidemic, Taiyuan made full use of various media methods such as TV, Internet, and Weibo to timely understand and grasp the latest epidemic prevention and control instructions of the Party Central Committee. By effectively combining the actual situation of this city, the spread of the potential epidemic situation is carefully analyzed and evaluated. Also, the strategies and programs for prevention and control are adjusted in real-time according to the monitored changes in the epidemic situation. After the epidemic prevention and control, it is found that the existing public health emergency monitoring system has the following shortcomings. The first is a longer response time. Generally, the average interval from the relevant information standard to the system creation time is too long. The second is the low utilization of information resources. Due to the decentralized management of information within the CDCP, monitoring and early warning information cannot be effectively integrated, and early warning cannot be played. In this epidemic, the Emergency Office of the Health Bureau opened a 24-hour duty phone, emergency network, and WeChat platform. Relevant emergency units are required to report to higher authorities within 24 hours after a crisis is discovered. Also, it cooperates with relevant responsible units for verification in time to ensure that relevant information can be communicated in time. The timeliness of the detection system has been greatly improved.

### 3.6. Material Reserve Management and Infrastructure Construction

The emergency material reserve is an important guarantee for the smooth handling of public health emergencies, and it is also a huge system project. After the outbreak of the COVID-19 epidemic, there is a shortage of masks, goggles, protective clothing, and some medical rescue equipment. It is related not only to the significant gap between demand and production reserves but also to the reasons for chaos in deployment, local conflicts of interest, and inefficient use. Although this situation is quickly alleviated, the shortage of medical and epidemic prevention materials in the early and middle stages of the epidemic has brought many hidden dangers to patient treatment, medical staff protection, and people's health protection. Therefore, it is necessary to attach great importance to the construction of medical emergency material reserves and guarantee systems required for major epidemics and disasters. The emergency material supply guarantee should be strengthened, and a complete set of material management system and unobstructed emergency material supply system should be established to ensure the storage and management of emergency materials.

The construction of the emergency rescue infrastructure for public health incidents should be strengthened. The open sharing mechanism for public data resources should be established in medical rescue and some departments such as laboratory testing, fire safety, road traffic, and credit management. The systematic and intelligent urban disaster emergency medical rescue should be rapidly realized. For example, in the process of responding to the epidemic, the special hospitals such as Huoshenshan Hospital and Leishenshan Hospital have been built in Wuhan. “Module hospitals” built in large convention centers and gymnasiums are all temporarily constructed and requisitioned sites. They are used to alleviate the problems caused by the lack of beds in conventional medical institutions, and it is a “realistic strategy.”

## 4. Conclusion

The construction of the public health emergency management system in Taiyuan has achieved remarkable results after the SARS in 2003. Emergency management capability has been greatly improved. In the COVID-19 epidemic prevention and control work, some results have been achieved, but some problems have been exposed. The discrete stochastic mathematical model and its analysis method proposed can be used as an important model framework for studying the epidemic development trend of Taiyuan or other similar cities (with a small number of cases but a large proportion of imported cases). In the case of a small proportion of imported cases, although maintaining intermittent population inflow will lead to a small-scale secondary outbreak, the transmission risk is low. By analyzing the problems highlighted in the prevention and control of the epidemic, the corresponding improvement measures are proposed. It is necessary to establish a sound coordination system of emergency health management and vigorously promote the construction of emergency health management institutions. Also, the preparation and implementation of prediction and early warning programs should be increased. The government should increase investment in funds, ensure emergency material reserves, increase laboratory equipment investment, and improve infrastructure construction. In addition, the construction of the public health talent team and the technology of testing personnel need to be improved. Thus, a public health emergency management system integrating management coordination system, plan system, emergency team building system, material reserve management, and other functions is formed. Improving the local government's public health emergency management capabilities is greatly significant for maintaining national social stability and economic development. For the specific emergency strategies of public health emergencies, this study has not explored in detail. The follow-up research can focus on discussing the emergency decision-making in combination with the prospect theory and other relevant theoretical basis.

## Figures and Tables

**Figure 1:** Schematic diagram of COVID-19 epidemic situation and prevention and control strategy model.

**Figure 2:** Public health emergency management system.

**Figure 3:** The onset time curve of confirmed cases of COVID-19 epidemic in Taiyuan.

**Figure 4:** Regional distribution of confirmed cases of COVID-19 epidemic in Taiyuan. Horizontal axes 1-6, respectively, represent Wanbailin District, Yingze District, Xinghualing District, Qingxu County, Xiaodian District, and unpublished source area.

**Figure 5:** Statistics on the nature of medical institutions in Taiyuan. Gov-med: governmental medical institutions; Non Gov-med: nongovernmental medical institutions; Soc-med: social medical institutions; Non Soc-med: nonsocial medical institutions; Gov-CHN: governmental Chinese medicine hospital; Non Gov-CHN: nongovernmental traditional Chinese medicine hospital.

**Figure 6:** Educational structure of health professional technicians in Taiyuan CDCP.

**Figure 7:** Positional title structure of health professional technicians in Taiyuan CDCP.

**Figure 8:** Total infrastructure area of CDCPs in Taiyuan.

**Figure 9:** Per capita area of infrastructure construction of CDCPs in Taiyuan.

**Table 1:** The medical and health institutions in Taiyuan.

Medical and health institution	Number of institutions	Number of beds
Public hospital	58	13296
Private hospital	43	5634
Community health service center (station)	126	657
Centers for Disease Control and Prevention	11	286
Specialized disease prevention and control institutions (institutes, stations)	1	150

## Data Availability

The data used to support the findings of this study are available from the corresponding author upon request.
